The article "Design and Analysis of a Flexible, Elastic, and Rope-Driven Parallel Mechanism for Wrist Rehabilitation" was published in 2020. Journal: Appl Bionics Biomech.

# Design and Analysis of a Flexible, Elastic, and Rope-Driven Parallel Mechanism for Wrist Rehabilitation

**DOI:** 10.1155/2020/8841400

**Published:** 2020-11-12

**Authors:** Zaixiang Pang, Tongyu Wang, Junzhi Yu, Shuai Liu, Xiyu Zhang, Dawei Jiang

**Affiliations:** ^1^School of Mechatronical Engineering, Changchun University of Science and Technology, Changchun, China; ^2^School of Mechatronical Engineering, Changchun University of Technology, Changchun, China; ^3^State Key Laboratory for Turbulence and Complex Systems, Department of Mechanics and Engineering Science, BIC-ESAT, College of Engineering, Peking University, Beijing, China

## Abstract

This paper proposes a bionic flexible wrist parallel mechanism to simulate human wrist joints, which is characterized by a rope-driven, compression spring-supported hybrid mechanism. Specifically, to realize the movement of the wrist mechanism, a parallel structure is adopted to support the mobile platform and is controlled by a cable, which plays the role of wrist muscles. Because the compression spring is elastic, it is difficult to directly solve inverse kinematics. To address this problem, the external force acting on the moving platform is firstly equivalent to the vector force and torque at the center of the moving platform. Then, based on inverse kinematic and static analyses, the inverse motion of the robot model can be solved according to the force and torque balance conditions and the lateral spring bending equation of the compression spring. In order to verify the proposed method, kinematics, statics, and parallel mechanism workspace are further analyzed by the software MATLAB. The obtained results demonstrate the effectiveness and feasibility of the designed parallel mechanism. This work offers new insights into the parallel mechanism with flexible joints in replicating the movements of the human wrist, thus promoting the development of rehabilitation robots and rope-driven technology to some extent.

## 1. Introduction

Stroke is known as apoplexy or cerebrovascular accident (CVA), and it is a persistent neurological deficit in the brain caused by acute cerebrovascular disease. After the onset of stroke, 85% of stroke patients may have motor dysfunction in one limb [1], i.e., hemiplegia. Clinical medicine proves that patients need scientific rehabilitation training to help patients recover when their joints have movement disorders or injuries [2]. Scientific rehabilitation refers to the personalized rehabilitation treatment of patients through formulating reasonable rehabilitation strategies and methods based on the traditional rehabilitation theory and combining the mechanical structure and robot characteristics so as to help patients with limb rehabilitation training. In traditional rehabilitation therapy, therapists perform one-to-one rehabilitation therapy on patients. This method is not only laborious and expensive but also difficult to guarantee the efficiency and intensity of training. The objective data is absent to evaluate the relationship between training parameters and rehabilitation effects. It is tough to optimize training parameters to obtain the best treatment plan [3]. With the widespread application of robotics in the field of rehabilitation medicine, robots for joint rehabilitation have emerged at the historic moment, and they have shown superiority over traditional treatments in clinical trials. The advantages of a rehabilitation robot as a partner or/and substitute physiotherapist lie in combining robot technology with clinical rehabilitation medicine. The rehabilitation robot can give full play to its advantages of being good at performing repetitive heavy labor, which can realize precise, automatic, and intelligent rehabilitation training to reduce the physiotherapist's heavy physical labor. The rehabilitation robot system can improve the efficiency of rehabilitation training. A physiotherapist can monitor the movement of several rehabilitation robots in real time and conduct rehabilitation training for several patients at the same time so as to reduce the number of physiotherapists and the cost of labor.

The article "Design and Analysis of a Flexible, Elastic, and Rope-Driven Parallel Mechanism for Wrist Rehabilitation" was published in 2020. Journal: Appl Bionics Biomech.

The rehabilitation robot system is more suitable for accurate and flexible rehabilitation training. It can adjust the motion parameters and force parameters applied to the patient in real time and accurately. Moreover, it makes the treatment more flexible and accurate. The rehabilitation robot system can monitor and record the changes of treatment parameters and patients' physiological signals in real time, which is more conducive to the quantitative analysis of doctors and convenient for the quantitative observation and comparison of patients to traditional medicine. At the later stage of rehabilitation treatment, the rehabilitation robot can be partially/completely separated from the physiotherapist under the guidance of the physiotherapist, and patients can enjoy similar treatment effects of the physiotherapist, thus avoiding serious property loss and huge economic burden to patients and society by wrong treatment [4–6].

At present, most upper limb rehabilitation robots are merely designed for patients' shoulder and elbow joints but they ignore the wrist joints even if the upper limb robots cover the wrist joint design when wearing; they only use it as a passive joint, and it does not provide driving force [7]. As a matter of fact, the human wrist joint exerts an enormous function on people's daily activities. To control the specific posture of the human hand, it is very important to enable the human hand to firmly interact with the external environment to lock the posture of the human hand, maintain the stability of the hand movement, and transfer the huge muscle force of the forearm into the hand which can realize the grasping of heavy objects. Moreover, the position of the human wrist joint also affects the movement of the human finger. For example, when the wrist joint is bent, it is very difficult to bend the movement of the human finger [8]. The movement of the wrist joint is mainly composed of flexion/extension and abduction/adduction of the wrist joint and is combined with internal/external rotation of the forearm [9]. Therefore, the research of the wrist rehabilitation robot mechanism is an important supplement to the upper limb exoskeleton rehabilitation robot [10]. Based on different mechanical structures and rehabilitation principles, numerous domestic and foreign scientific research institutions and medical institutions have proposed a variety of wrist rehabilitation robot structures. Some examples of wrist joint rehabilitation robots are the RiceWrist [11, 12], the CRAMER [13], the InMotion's robot [14], and the SUE's rehabilitation robot [15], which can be seen as 2-degree of freedom (DOF) forearm/wrist rehabilitation robots and 3-DOF wrist rehabilitation robots [16–18]. By analyzing the existing wrist rehabilitation robots, it is known that the structure of the robot is mostly a tandem mechanism. Most of the existing wrist rehabilitation robots are series mechanisms, which are composed of several basic mechanisms with a single degree of freedom in sequence, forming a series combination. However, there are relatively few parallel mechanisms, for example, the parallel wrist rehabilitation robot (PWRR) [19], orthosis for wrist rehabilitation [20], and design of parallel wrist rehabilitation robot based on series elastic actuators [21]. There are also problems such as inability to fit the actual motion trajectory of the wrist, insufficient recovery effect, prone to deadlock, inaccurate motion control, and difficulty in coordinating with other upper limb rehabilitation robots to achieve coordinated training of upper limb joints.

The article "Design and Analysis of a Flexible, Elastic, and Rope-Driven Parallel Mechanism for Wrist Rehabilitation" was published in 2020. Journal: Appl Bionics Biomech.

In order to solve the above problems, a flexible human wrist parallel mechanism driven by a cable and compressed by springs is proposed to imitate the human muscle-tendon drive method, which is used to replicate the human wrist joint and has the advantages of a series mechanism and a parallel mechanism. Compared with the traditional series mechanism, the parallel mechanism has the advantages of small motion inertia, high bearing capacity, and fast dynamic response [22]. Besides the above advantages, the rope-driven parallel mechanism also has the advantage of large working space, high accuracy, and the characteristics of remote driving [23]. The mechanism is rope-driven to avoid the inertial impact of rigid rods, which can better meet the patients' requirements for the flexibility, safety, and comfort of the rehabilitation mechanism. At the same time, the rotation center of the mechanism coincides with the rotation center of the joint, which can effectively avoid secondary injuries to patients.

The purpose of this paper is to propose a bionic flexible wrist parallel mechanism driven by rope and supported by compression spring. The mechanism consists of three ropes and one cylindrical compression spring. The compression spring is used to simulate the supporting structure of the human wrist and support the mobile platform to complete the movement of the wrist, and the rope is used to simulate the wrist muscles to drive and control the parallel mechanism to realize the wrist flexion/extension and abduction/adduction motions. To capture the bending characteristics of the spring in the flexible wrist parallel mechanism, a system dynamic modeling method is proposed based on flexible vibration. Furthermore, the kinematic and static mechanics models of the flexible wrist parallel mechanism are developed, investigated, and analyzed due to force/torque equilibrium conditions and the lateral bending equation of compression spring. Besides, the correctness of the solution which is generated from the flexible wrist parallel mechanism is verified by numerical simulations.

The rest of this paper are organized as follows. In Section 2, we analyze the wrist joints of the human body and design a mechanical system model of the wrist joints based on the anatomy of the human wrist mechanism and the study of the movement mechanism and range of motion. In Section 3, the system dynamic model of the flexible parallel mechanism driven by the cable is established based on the flexible vibration factors. In Section 4, the inverse kinematic and static analyses of the flexible parallel mechanism driven by the cable are carried out by considering the spring lateral bending equation, and the correctness of the solution is verified by simulation analysis. In Section 5, in order to obtain better motion performance, the working space of the parallel mechanism is analyzed via numerical simulations. Finally, Section 6 gives concluding remarks.

## 2. Mechanical Structure Design

During daily activities, upper limbs mainly perform actions such as eating, holding things, and touching the head. The wrist joint not only owns a high frequency of movement but also refers to the part of the human body's upper limbs that bears the most load during support and push-pull movements. In this paper, we propose a bionic flexible rope-driven wrist parallel joint structure, which is mainly a device for midterm semiactive rehabilitation training and postactive rehabilitation training for stroke patients who have mobility in the wrist. During rehabilitation training, the patients need to hold the adjustable handle which lies at the end of the bionic flexible rope-driven wrist parallel joint structure, and then the upper limb will do the corresponding rehabilitation training with the parallel mechanism.

The article "Design and Analysis of a Flexible, Elastic, and Rope-Driven Parallel Mechanism for Wrist Rehabilitation" was published in 2020. Journal: Appl Bionics Biomech.

The movement of the wrist includes 2-DOFs which are flexion/extension and abduction/adduction. When the 2-DOFs are combined with pronation and supination movements around the long axis of the forearm, the wrist joint is increased the third degree of freedom (pronation and supination) [24, 25]. During the rehabilitation training, the wrist does not need a lot of force. In the meantime, the amplitude of the passive flexion and extension of the wrist in the 3-DOFs is small. During rehabilitation training, the wrist can be fully trained through another 2-DOF exercise [26]. Thus, in order to simplify the structure and reduce the control difficulty under the premise of ensuring basic functions, this paper will not design passive flexion and extension exercises, which can reduce the complexity of the mechanical structure and maximize the restoration of the wrist joints of the human upper limbs. Since the carpal palmar ligament is relatively tough, the movement of the extension is restricted, and the radial styloid process is low, and it will abut with most of the horns during the abduction. Therefore, the abduction of the wrist is much smaller than the adduction. During human daily activities, the maximum range of flexion/extension of the human upper limb is 150°, while the abduction/adduction is 50°. The wrist complex and the freedom of movement of the wrist joint are shown in Figure 1.

According to the physiological structure characteristics of the wrist joint and the wrist muscle-skeletal biological coupling, the movement pattern of the wrist joint is extracted by analyzing the movement mechanism of the wrist. The ulnar carpi flexor and the radial carpi flexor are simplified, and the palmaris longus is a bundle of muscles to achieve flexion/flexion of the wrist joint. It simplifies the ulnar carpi flexor and ulnar carpi extensor and radial carpi flexor. The palmar long muscle and radial extensor muscles perform a wrist abduction/adduction motion for a bundle of muscles, respectively.

The article "Design and Analysis of a Flexible, Elastic, and Rope-Driven Parallel Mechanism for Wrist Rehabilitation" was published in 2020. Journal: Appl Bionics Biomech.

This paper proposes a bionic flexible rope-driven wrist parallel mechanism. The wrist structure adopts the hand-wrist-forearm connection method. The front and back parts of the wrist are connected by a cylindrical compression spring. The cylindrical compression spring is utilized to simulate the human wrist joint. There are three sets of cable mechanisms around the mechanism. Each group of the cable mechanisms contains 120 degrees apart to simulate wrist muscles to complete the drive control of the wrist. Each cable mechanism is equipped with a power source of the base. The design of the flexible parallel mechanism is bionic to the human wrist. The fixed ring is equivalent to the human radius and ulna complex. The moving ring can be viewed as a human metacarpal. The driving cables and springs correspond to the muscles and ligaments around the human wrist, and they provide the corresponding kinetic energy and support for the movements of the radial and middle wrist joints. The parallel mechanism drives three cables through three servo motors to achieve wrist flexion/extension and abduction/adduction motions. This method ensures that the mechanism enhances the stability of the mechanism while completing the adduction and abduction, flexion, and straightening actions and can satisfy the motion range of the wrist at different angles. Consequently, the mechanism can achieve flexion/extension and abduction/adduction of the wrist joint. As shown in Figure 2, the flexible parallel joint of the wrist driven by the cable is mainly composed of an adjustable handle, a flexible parallel mechanism, and a forearm fixing.

The most important point of the exoskeleton rehabilitation robots matches with human joints. The distance between the axis of each patient's fist and the flexion/extension axis of the wrist has a certain difference, and some patients with severe hemiplegia need to fix their fingers to the handle with bandages. In the meantime, the distance between the two axes will be more significantly deviated. Therefore, the bionic flexible rope-driven wrist parallel mechanism can adjust the distance between the two axes according to different patients, which can help patients to complete comfortable rehabilitation training while avoiding secondary injuries to the patients. As illustrated in Figure 3, the adjustable device consists of a slide rail, a slider, and a handle, which can realize the precise adjustment of the distance *L* between the two axes.

The flexible parallel mechanism is depicted in Figure 4, which is the core of a bionic flexible cable-driven wrist parallel mechanism. The mechanism consists of a compression spring, three cables, a moving ring, and a fixed ring. Because the bionic flexible rope-driven wrist parallel mechanism needs rehabilitation training of wrist flexion/extension and adduction/abduction deviation, three cable restraints are distributed on the moving ring and the fixed ring at 120° intervals so that it can simulate wrist muscle movements. Each cable restraint device is composed of a bracket and a restraining wheel. A cable restraint device on the fixing ring is taken as an example shown in Figure 5. The bracket can achieve relative rotation with the fixed ring about the *r*_1_ axis, and the restraint wheel can achieve relative rotation with the bracket about the *r*_2_ axis.

The article "Design and Analysis of a Flexible, Elastic, and Rope-Driven Parallel Mechanism for Wrist Rehabilitation" was published in 2020. Journal: Appl Bionics Biomech.

If no device is added to the moving ring and fixed ring, as shown in Figure 6, the flexible parallel mechanism will consume the cable length due to the mechanical structure during movement. And it will have a large friction coefficient, which will bring a lot of noise and reduce the life of the device.  Figure 7 shows that these issues have been resolved with the addition of the cable restraint and the blue part of the cable in comparison. It can be found that the cable restraint device is added; the cable always maintains the shortest length in the flexible parallel mechanism, which ensures the consistency between the theoretical model and the actual device. It is essential to realize the precise control of the rehabilitation robot. Theoretically, the cable restraint device only needs to make the restraint wheel rotate relative to the bracket to meet the precise control requirements of the robot. However, considering that the patient applies a certain load during the training process, a slight misalignment between the moving ring and the fixed ring of the flexible parallel mechanism is unavoidable. Therefore, the degree of freedom of rotation of the bracket around the ring is increased to avoid errors caused by misalignment. However, the patient needs to apply a certain load during the rehabilitation training process, which will inevitably lead to a slight misalignment between the moving ring and the fixed ring of the flexible parallel mechanism. Therefore, errors caused by misalignment are avoided by increasing the degree of freedom of rotation of the bracket around the ring.

Figure 8 shows that the forearm fixing part is a conical structure as a whole. The purpose of the forearm fixing part is to fit the curvature of the forearm of the human body and improve the wearing comfort. The path and initial length of the cable are determined by cable ties and conduit.

## 3. Flexible Vibration Factors of the System Dynamic Model

The rope-driven parallel mechanism converts the movement state and force of the driver with the driving cable as the medium and converts it into the movement state and force of the end effector. The rope-driven parallel mechanism is a type of parallel mechanism that uses a cable instead of a rigid rod drive [27, 28]. This mechanism is different from a rigid rod. The cable can only provide tension; therefore, the cable should always be kept under tension in the working space of the mechanism. Once the cable loosens, the structure of the mechanism will collapse. In the rope-driven mechanism, the end effector is connected to a fixed platform via using several cables, and the end effector is driven to move to a desired position and direction by adjusting the cable length or cable tension [29]. The structure determines that the rope-driven parallel mechanism has the advantages of reconfigurability, low inertia, fast maneuverability, large working space, high load/mass ratio, and remote driving.

The article "Design and Analysis of a Flexible, Elastic, and Rope-Driven Parallel Mechanism for Wrist Rehabilitation" was published in 2020. Journal: Appl Bionics Biomech.

This paper presents a simplified bionic wrist parallel mechanism that simulates a human upper limb wrist joint with a cylindrical compression spring and three cables to simulate wrist muscles. The mechanism needs redundant force to achieve the force closing the parallel mechanism because the cable can only exert unidirectional tension and cannot generate thrust. In order to achieve a rope-driven parallel mechanism with *η* degrees of freedom and obtain a positive cable tension, there must be *η* + 1 cables as driving elements. Due to the variable length of the spring, it can bear both pressure and tensile force. The introduction of the spring into the parallel cable mechanism can provide a driven force for the cable traction parallel mechanism that can change in size and direction as the end effector moves. Selecting the proper position and parameters (i.e., initial length and stiffness coefficient) of the spring can reduce the number of actuators required by the parallel mechanism for cable traction and form a rope-driven mechanism with the same number of degrees of freedom, making the rope-driven parallel mechanism control more simple [30, 31]. Hence, in the designed parallel mechanism, only three cables driving the platform with a 120° distribution are required to achieve 2-DOFs. The three cables are of equal arc length on the moving platform and the fixed platform.

The schematic diagram of the designed bionic flexible wrist parallel mechanism is shown in Figure 9. It is mainly composed of four parts: base, moving platform, cable, and spring. The fixed part of the mechanism is the fixed platform. The global coordinate system *OXYZ* of the parallel mechanism is set on the fixed platform. The origin *O* of the coordinate system is located at the geometric center of the fixed platform, where the *Y*-axis is in the direction of *OP*_1_, and the *X*-axis and the *Y*-axis are perpendicular to each other. Determine the *Z*-axis by the right-hand rule; the direction of the *Z*-axis is upward and perpendicular to the plane where the fixed platform is located. The moving platform is a nonfixed part of the parallel mechanism, which is driven by three motors driving three cables. The local coordinate system *oxyz* of the flexible parallel mechanism is defined on the moving platform. The origin *o* of the coordinate system is located at the geometric center of the top of the moving platform spring, the *Y*-axis direction is along the *oQ*_1_ direction, the *x*-axis direction is perpendicular to the *y*-axis, and the *z*-axis direction is perpendicular to the plane where the moving platform is located. The cable in the parallel mechanism is composed of three flexible cables with negligible mass and diameter. One end of each driving cable is fixed to the point *Q*_*i*_(*i* = 1, 2, 3) on the moving platform. The other end is fixed to the output end of the drive motor, and the cable passes through the fixed platform through the point *P*_*i*_. In the initial state (i.e., natural state without load), $\vec{{OP}_{i}}$ and $\vec{{oQ}_{i}}$ are in the same direction, while *P*_*i*_ and *Q*_*i*_ are distributed at a medium distance in a circle with a radius of |*OP*_*i*_| = *a* and |*oQ*_*i*_| = *b*, respectively. *T*_*i*_ represents the pulling force of the cable, the cable length between *P*_*i*_ and *Q*_*i*_ is *l*_*i*_, and the pulling direction of each cable is the unit vector along the cable direction which is *u*_*i*_. The spring is connected between the fixed platform and the moving platform and uses the generated force or torque generated by it to support the robot wrist load and realize head movement.

The article "Design and Analysis of a Flexible, Elastic, and Rope-Driven Parallel Mechanism for Wrist Rehabilitation" was published in 2020. Journal: Appl Bionics Biomech.

Figure 10 shows the force and torque balance system in the spring bending plane and does not show the *δ*_*s*_ variable, since the moving platform in the parallel mechanism will produce two motion angles *δ*_*s*_ and *δ*_*p*_ under the action of the tension of three ropes. *δ*_*s*_ is used to describe the angle to which the moving platform bends, and *δ*_*p*_ is utilized to describe the bending angle of the moving platform. When the parallel mechanism is stationary, the tension in all ropes can be transformed into the force and moment in the plane *Ost*; otherwise, the spring will not bend in the plane. Therefore, the tension of the rope can be equivalent to two mutually perpendicular forces *F*_1_ and *F*_2_ in the *Ost* plane and the moment *M* passing through the *o* point and perpendicular to the *Ost* plane. Assuming that the moving platform is not affected by other external forces, the moving platform can be regarded as a point with mass *m* at point *o*. When *δ*_*s*_ is given, the only corresponding *Ost* plane will be determined, and Figure 10 shows the *Ost* plane which is uniquely determined.

There is a curve between point *O* and point *o* in Figure 10. At point *O*, the tangent direction of the curve is perpendicular to the plane on which the base is located. At point *o*, the tangent direction of the curve is perpendicular to the plane on which the moving platform is located. In order to analyze the system, it defined that the spring only bends in the same plane, and the torsional strength of the spring is very large. So it can be considered that the moving platform will not rotate about the *z*-axis direction in the local coordinate system *oxyz*. At the same time, the rectangular coordinate system *Ost* is introduced in the *Ooo*′ plane (*o*′ is the projection of the center point *o* of the moving platform on the plane *OXY* where the fixed platform is located). The origin of this coordinate system is the same as the origin *O* of the global coordinate system *OXYZ*, the *t*-axis coincides with the *Z*-axis, and the *s*-axis is along the direction of the ray *Oo*′.

According to the set situation, the structure of the moving platform can be quantified into four parameters: *δ*_*s*_ is the angle between the *s*-axis and the *X*-axis and represents the bending direction of the spring; *δ*_*p*_ is the included angle between the plane where the fixed platform is located and the plane where the moving platform is located and means the amplitude of spring bending; *t*_0_ is the vertical distance between the origin of the moving platform and the plane of the fixed platform. *s*_0_ is the distance between *O* and *o*′ of the origin of the platform. Parameters *δ*_*s*_ and *δ*_*p*_ are exploited to describe the attitude of the moving platform in the global coordinate system *OXYZ*, while parameters *t*_0_ and *s*_0_ are utilized to describe the position of the moving platform in the global coordinate system *OXYZ*. One of the parameters *t*_0_ and *s*_0_ is independent merely as the result of the lateral bending characteristic equation of the flexible spring. Therefore, for the above four parameters, three of them are independent. In order to lose fraction, parameter *s*_0_ is regarded as a subordinate parameter of the other three parameters. Parameter *s*_0_ can be solved by *δ*_*s*_, *δ*_*p*_, and *t*_0_, which is generally regarded as an accompanying motion determined by the other three parameters. The number of degrees of freedom of the mechanism is the number of independent coordinates defining the configuration of the mechanism. Thus, the mechanism has only 3-DOFs *δ*_*s*_, *δ*_*p*_, and *t*_0_. The attitude of the moving platform in the mechanism can be described by *δ*_*s*_ and *δ*_*p*_; the attitude transformation matrix of the moving platform can be obtained when its value is given.

The article "Design and Analysis of a Flexible, Elastic, and Rope-Driven Parallel Mechanism for Wrist Rehabilitation" was published in 2020. Journal: Appl Bionics Biomech.

The dynamic model of the system is constructed by considering only the flexible vibrations of the spring (i.e., axial flexible vibration and radial flexible vibration). To describe the geometric relationship between different basis points, the direction cosine matrix must be extended [32, 33]. The direction cosine matrix is extended into a square matrix with the 4th order by means of vector diameter to realize the transformation between different bases. According to the number, 1 is added as the 4th coordinate to become the homogeneous coordinate of the vector, except for three projections of the vector onto the basis vector. As an extension of the function of the direction cosine matrix to deal with the rotation of the rigid body, the homogeneous coordinate transformation matrix can deal with the varying process of the rotation and movement of the rigid body. In this case, the means of using the homogeneous coordinate transformation matrix is exactly the same as the direction cosine matrix for the coordinate transformation.

Under the global coordinate system *OXYZ*, the homogeneous coordinate transformation matrix at point *P*_*i*_(^0^*p*_1_, ^0^*p*_2_, ^0^*p*_3_) on the fixed platform can be expressed as

(1) p01=0,a,0,1T,p02=−32a,−12a,0,1T,p03=32a,−12a,0,1T.

Under the local coordinate system *oxyz*, the homogeneous coordinates of point *Q*_*i*_(^0^*q*_1_, ^0^*q*_2_, ^0^*q*_3_) on the moving platform can be seen as

(2) q01=0,b,0,1T,q02=−32b,−12b,0,1T,q03=32b,−12b,0,1T.

By using the coordinate matrix formula of the finite rotation tensor, the finite rotation matrix $\underline{A}$ from the local coordinate system to the global coordinate system is obtained, that is,

(3) $$\begin{array}{c} \underline{A}=\cos\delta_{p}\underline{E}+\left(1-\cos\delta_{p}\right){\underline{\omega }\underline{\omega }}^{T}+\sin\delta_{p}\underline{\omega }. \end{array}$$

Let

(4) $$\begin{array}{c} p_{1}=-\sin\delta_{s},\\ p_{2}=\cos\delta_{s},\\ p_{3}=0. \end{array}$$

From formula $\underline{\omega }=\left[\begin{array}{ccc} -\sin\delta_{s} & \cos\delta_{s} & 0 \end{array}\right]$, $\hat{\underline{\omega }}$ is the antisymmetric coordinate matrix of $\underline{\omega }$; the details can be seen as follows. $\underline{E}$ is the unit vector matrix.

(5) $$\begin{array}{c} \underline{\hat{\omega }}=\left[\begin{array}{ccc} 0 & 0 & \cos\delta_{s}\\ 0 & 0 & \sin\delta_{s}\\ -\cos\delta_{s} & -\sin\delta_{s} & 0 \end{array}\right]. \end{array}$$

The finite rotation matrix is obtained as follows:

(6) $$\begin{array}{c} \underline{A}=\cos\delta_{p}\underline{E}+\left(1-\cos\delta_{p}\right)\left[\begin{array}{c} -\sin\delta_{s}\\ \cos\delta_{s}\\ 0 \end{array}\right]\left[\begin{array}{ccc} -\sin\delta_{s} & \cos\delta_{s} & 0 \end{array}\right]+\sin\delta_{p}\left[\begin{array}{ccc} 0 & 0 & \cos\delta_{s}\\ 0 & 0 & \sin\delta_{s}\\ -\cos\delta_{s} & -\sin\delta_{s} & 0 \end{array}\right]=\left[\begin{array}{ccc} \cos\delta_{p}+\left(1-\cos\delta_{p}\right)\sin^{2}\delta_{s} & -\left(1-\cos\delta_{p}\right)\sin\delta_{s}\cos\delta_{s} & \sin\delta_{p}\cos\delta_{s}\\ -\left(1-\cos\delta_{p}\right)\sin\delta_{s}\cos\delta_{s} & \cos\delta_{p}+\left(1-\cos\delta_{p}\right)\cos^{2}\delta_{s} & \sin\delta_{p}\sin\delta_{s}\\ -\sin\delta_{p}\cos\delta_{s} & -\sin\delta_{p}\sin\delta_{s} & \cos\delta_{p} \end{array}\right]. \end{array}$$

Thus, from the local coordinate system to the global coordinate system, the homogeneous coordinate transformation matrix ^*o*^*T*_*o*_ can be generalized as

(7) Too=t^11t^12t^13s0cosδst^21t^22t^23s0sinδst^31t^32t^33t00001,

where

(8) $$\begin{array}{c} {\hat{t}}_{11}=\sin^{2}\delta_{s}+\cos^{2}\delta_{s}\cos\delta_{p},\\ {\hat{t}}_{12}=\left(\cos\delta_{p}-1\right)\cos\delta_{s}\sin\delta_{s},\\ {\hat{t}}_{13}=\sin\delta_{p}\cos\delta_{s},\\ {\hat{t}}_{21}=\left(\cos\delta_{p}-1\right)\sin\delta_{s}\cos\delta_{s},\\ {\hat{t}}_{22}=\cos^{2}\delta_{s}+\cos\delta_{p}\sin^{2}\delta_{s},\\ {\hat{t}}_{23}=\sin\delta_{p}\sin\delta_{s},\\ {\hat{t}}_{31}=-\sin\delta_{p}\cos\delta_{s},\\ {\hat{t}}_{32}=-\sin\delta_{p}\sin\delta_{s},\\ {\hat{t}}_{33}=\cos\delta_{p}. \end{array}$$

The article "Design and Analysis of a Flexible, Elastic, and Rope-Driven Parallel Mechanism for Wrist Rehabilitation" was published in 2020. Journal: Appl Bionics Biomech.

## 4. Inverse Kinematic and Static Analyses

In the inverse kinematic analysis of the system, the attitude matrix of the moving platform required by the robot is given, and the length *ρ*_*i*_ of the rope is required to be solved. Let $X={\left[\begin{array}{ccc} \delta_{s}, & \delta_{p}, & t_{0} \end{array}\right]}^{T}\in R^{3}$ and $q={\left[\begin{array}{ccc} \rho_{1}, & \rho_{2}, & \rho_{3} \end{array}\right]}^{T}\in R^{3}$; the relationship between *X* and *q* can be seen as

(9) $$\begin{array}{c} q=f\left(x\right),f:R^{3}⟶R^{3}. \end{array}$$

If *s*_0_ is obtained from *x*, ^*o*^*T*_*o*_ can be completely determined and the lengths of each rope are obtained from *l*_*i*_ = ‖^*o*^*a*_*i*_ − ^*O*^*T*_*o*_^*o*^*b*_*i*_‖. Since *s*_0_ is an accompanying motion that occurs when the spring is bent sideways. The numerical value cannot be set arbitrarily but generated by the force applied on the spring. The force on the spring is caused by the pull of the three ropes and the weight of the load [34, 35]. Therefore, in order to solve the problem, the inverse kinematics and statics of the parallel rope mechanism will be combined for analysis.

### 4.1. Spring Static Equation

In this paper, all the rope tension is converted into equal force and equivalent torque applied to the center of the spring top. All the rope tension can be converted into force and torque in the spring bending plane*Ost*; otherwise, the spring is not bending in the plane. As shown in Figure 10, the tension of all ropes can be equivalent to two mutually perpendicular forces *F*_1_ and *F*_2_ in the *Ost* plane and one moment *M* perpendicular to *Ost* of the spring bending plane through point *o*. Then, the kinematics of the mechanism is solved by combining the lateral bending equation of the spring with the balance equation of force and torque applied on the moving platform.

The lateral bending problem of the spiral compression spring can be solved by analyzing the elastic bar. The flexible spring will bend under the action of two forces *F*_1_ and *F*_2_ and a torque *M*. Assume that the bionic flexible parallel mechanism driven by rope can be bent in a small angle range and only the linear curve of the spring is considered. For any section of the spring, the linear equation of small bending can be generalized as

(10) $$\begin{array}{c} \beta \frac{d^{2}s}{{dt}^{2}}=M+F_{2}\left(s_{0}-s\right)+F_{1}\left(t_{0}-t\right). \end{array}$$

The initial conditions for connecting the fixed end of the platform and the free end of the moving platform can be obtained as follows:

(11) $$\begin{array}{c} s\left(0\right)=0,\\ s^{\prime }\left(0\right)=0,\\ s\left(t_{0}\right)=s_{o},\\ s^{\prime }\left(t_{0}\right)=\tan\delta_{p}, \end{array}$$

where

(12) $$\begin{array}{c} s^{\prime }=\frac{d_{s}}{d_{t}}. \end{array}$$

According to equations (10) and (11), the following two equations which can be defined as and can be derived as a function of

(13) $$\begin{array}{c} F_{1}=D_{1}s_{0}+E_{1}, \end{array}$$

(14) $$\begin{array}{c} M=D_{2}s_{0}+E_{2}, \end{array}$$

where.

(15) $$\begin{array}{c} D_{1}=-\frac{a_{2}c_{1}-a_{1}c_{2}}{a_{2}b_{1}-a_{1}b_{2}},\\ E_{1}=-\frac{a_{2}d_{1}-a_{1}d_{2}}{a_{2}b_{1}-a_{1}b_{2}},\\ D_{2}=-\frac{b_{2}c_{1}-b_{1}c_{2}}{a_{1}b_{2}-a_{2}b_{1}},\\ E_{2}=-\frac{b_{2}d_{1}-b_{1}d_{2}}{a_{1}b_{2}-a_{2}b_{1}},\\ a_{1}=1-\cos\left(\sqrt{\frac{F_{2}}{\beta }}t_{0}\right),\\ b_{1}=\sqrt{\frac{\beta }{F_{2}}}\sin\left(\sqrt{\frac{F_{2}}{\beta }}t_{0}\right)-t_{0}\cos\left(\sqrt{\frac{F_{2}}{\beta }}t_{0}\right),\\ c_{1}=-F_{2}\cos\left(\sqrt{\frac{F_{2}}{\beta }}t_{0}\right),\\ d_{1}=0,\\ a_{2}=\sqrt{\frac{F_{2}}{\beta }}\sin\left(\sqrt{\frac{F_{2}}{\beta }}t_{0}\right),\\ b_{2}=\cos\left(\sqrt{\frac{F_{2}}{\beta }}t_{0}\right)+t_{0}\sqrt{\frac{F_{2}}{\beta }}\sin\left(\sqrt{\frac{F_{2}}{\beta }}t_{0}\right)-1,\\ c_{2}=F_{2}\sqrt{\frac{F_{2}}{\beta }}\sin\left(\sqrt{\frac{F_{2}}{\beta }}t_{0}\right),\\ d_{2}=-F_{2}\tan\delta_{p}, \end{array}$$

where *β* represents the flexural stiffness of the spring after compression. Owing to the spring bending stiffness *β*_0_ and spring length (the initial length *ρ*_0_ and the compressed length *t*_0_), *β* can be expressed as follows:

(16) $$\begin{array}{c} \beta =\beta_{0}\frac{t_{0}}{\rho_{0}}. \end{array}$$

In this paper, *t*_0_ is an approximate length of the compressed spring. In practice, the compressed length of the spring is equal to *t*_0_ when the spring is not bent at all (*δ*_*p*_ = 0). If *δ*_*p*_ ≠ 0, *t*_0_ can be approximated through the compressed spring length since the spring used in this paper only produces a small amount of deformations in practical applications. Therefore, the variable *F*_2_ can be approximately computed by Hooke's law as

(17) $$\begin{array}{c} F_{2}\approx K\left(\rho_{0}-t_{0}\right), \end{array}$$

where *K* represents the stiffness coefficient of the spring and *ρ*_0_ denotes the original length of the spring.

The article "Design and Analysis of a Flexible, Elastic, and Rope-Driven Parallel Mechanism for Wrist Rehabilitation" was published in 2020. Journal: Appl Bionics Biomech.

### 4.2. Equilibrium Equations of Force and Torque

In general, assume that all ropes must be able to generate tension to achieve the equilibrium of the moving platform without being affected by other external forces. In this case, the moving platform can be regarded as a particle of mass *m* at point *o* at the center of the moving platform. Therefore, the equilibrium equation of force and torque of the moving platform can be obtained as follows:

(18) ∑i=13TiOui+F=0,∑i=13rOi×TiuOi+M=0.

It follows that

(19) F=F1cosδS,F1sinδS,F−mgT,M=−Msinδs,Mcosδs,0T,uOi=aOi−TooboiaOi−Tooboi,rOi=ROo×oQi→.

There are 7 unknown variables in equation (18), namely, *T*_1_, *T*_2_, *T*_3_, *F*_1_, *F*_2_, *M*, and *s*_0_. By eliminating *T*_1_, *T*_2_, and *T*_3_, an equation with only four unknown parameters can be obtained; the details can be seen as the following unknown variables *F*_1_, *F*_2_, *M*, and *s*_0_. According to the compression and bending equations of the spring, the three unknowns *F*_1_, *F*_2_, and *M* can be solved by equations (14), (16), and (17) and *T*_1_, *T*_2_, an *T*_3_ in terms of *s*_0_.

Given or *s*_0_sin*δ*_*p*_ + *t*_0_(cos*δ*_*p*_ − 1) ≠ 0 and $\theta_{s}\neq k\pi /2\left(\begin{array}{cccc} 0, & 1, & 2, & \cdots \end{array}\right)$, then

(20) $$\begin{array}{c} 2b\sin\delta_{s}\sin\delta_{p}{F_{2}}^{\prime }s_{0}^{2}+2b\left(\sin\delta_{s}\sin\delta_{p}t_{0}F_{1}+\sin\delta_{s}\cos\delta_{p}t_{0}F_{2}^{\prime }\right)s_{0}+2b\left(\sin\delta_{s}\sin\delta_{p}M+\frac{1}{2}a\sin\delta_{p}\cos2\delta_{s}F_{2}^{\prime }\right)s_{0}+b\left(2t_{0}^{2}\sin\delta_{s}\cos\delta_{p}-ab\sin\delta_{s}\sin^{2}\delta_{p}+a\sin\delta_{p}\cos2\delta_{s}t_{0}\right)F_{1}-ab\sin\delta_{s}\sin\delta_{p}\left(a-b\cos\delta_{p}\right)F_{2}^{\prime }-2t_{0}\sin\delta_{s}\left(a-b\cos\delta_{p}\right)M=0. \end{array}$$

In equation (20), *F*_1_, *F*_2_′, *M*, and *s*_0_ are unknown variables. *F*_2_′ can be obtained by *t*_0_, and *F*_1_ and *M* can be represented by the linear function of *s*_0_, respectively. Thus, the value of *s*_0_ can be obtained by solving equation (20). And if the posture of the moving platform is determined, unknown quantities ^*o*^*T*_*o*_, *l*_*i*_, and *T*_*i*_ can be obtained.

The article "Design and Analysis of a Flexible, Elastic, and Rope-Driven Parallel Mechanism for Wrist Rehabilitation" was published in 2020. Journal: Appl Bionics Biomech.

In the proceeding of analyzing the spring lateral bending problem, *F*_1_ and *M* can be expressed as functions of *s*_0_, and equations (14) and (16) can be substituted into equation (20) which can be obtained a quadratic equation of *s*_0_, namely,

(21) $$\begin{array}{c} {As}_{0}^{2}+{Bs}_{0}+C=0, \end{array}$$

where

(22) $$\begin{array}{c} A=2b\sin\delta_{p}\sin\delta_{s}\left(F_{2}^{\prime }+t_{0}D_{1}+D_{2}\right),\\ B=\left(2{bt}_{0}^{2}\cos\delta_{p}\sin\delta_{s}-{ab}^{2}\sin^{2}\delta_{p}\sin\delta_{s}+{abt}_{0}\sin\delta_{p}\cos2\delta_{s}\right)D_{1}+2{bt}_{0}\sin\delta_{s}\left(F_{2}^{\prime }\cos\delta_{p}+E_{1}\sin\delta_{p}\right)-2t_{0}\sin\delta_{s}\left(a-b\cos\delta_{p}\right)D_{2}+2b\sin\delta_{p}\left(E_{2}\sin\delta_{s}+\frac{1}{2}aF_{2}^{\prime }\cos2\delta_{s}\right),\\ C=\left(2{bt}_{0}^{2}\cos\delta_{p}\sin\delta_{s}-{ab}^{2}\sin^{2}\delta_{p}\sin\delta_{s}+{abt}_{0}\sin\delta_{p}\cos2\delta_{s}\right)E_{1}-ab\sin\delta_{p}\sin\delta_{s}\left(a-b\cos\delta_{p}\right)F_{2}^{\prime }-2t_{0}\sin\delta_{s}\left(a-b\cos\delta_{p}\right)E_{2}. \end{array}$$

The main purpose is to find *s*_0_ ∈ *R* ≥ 0 in this paper. Once *s*_0_ is known, all the unknown variables can be found out.

If *a* ≠ *b* or *s*_0_sin*δ*_*p*_ + *t*_0_(cos*δ*_*p*_ − 1) ≠ 0 holds, the following equation can be obtained:

(23) $$\begin{array}{c} \cos\delta_{s}\left(T_{1}^{\prime }-\frac{1}{2}\left(T_{2}^{\prime }+T_{3}^{\prime }\right)\right)+\frac{\sqrt{3}}{2}\sin\delta_{s}\left(T_{2}^{\prime }-T_{3}^{\prime }\right)=0. \end{array}$$

When equation (23) is not valid, *a* ≠ *b* and *s*_0_sin*δ*_*p*_ + *t*_0_(cos*δ*_*p*_ − 1) = 0 are required. In this case, it is only true when *δ*_*p*_ = 0, but since it represents that the wrist has not done any bending motion, the research is of little significance. Assume that *δ*_*p*_ ≠ 0; we ensure that equation (23) is always true.

The article "Design and Analysis of a Flexible, Elastic, and Rope-Driven Parallel Mechanism for Wrist Rehabilitation" was published in 2020. Journal: Appl Bionics Biomech.

When *δ*_*s*_ = *kπ*/2, *δ*_*s*_ has four special points in the interval $\left[\begin{array}{cc} 0, & 2\pi \end{array}\right]$, that is,$\delta_{s}=\begin{array}{cccc} 0, & \pi /2, & \pi , & 3\pi /2 \end{array}$. In this paper, only the case of *δ*_*s*_ = *π* pairs is deduced, and other special cases are similar to the derivation process.

When *δ*_*s*_ = *π*, it can be known that *T*_1_′ = (*T*_2_′ + *T*_3_′)/2, and equations (6), (10), and (14) are simplified to

(24) $$\begin{array}{c} s_{0}\left({T_{1}}^{\prime }+{T_{2}}^{\prime }+{T_{3}}^{\prime }\right)-\frac{\sqrt{3}}{2}\left(a-b\cos\delta_{p}\right)\left({T_{2}}^{\prime }-{T_{3}}^{\prime }\right)+F_{1}=0,\\ t_{0}\left({T_{1}}^{\prime }+{T_{2}}^{\prime }+{T_{3}}^{\prime }\right)-\frac{\sqrt{3}}{2}b\sin\delta_{p}\left({T_{2}}^{\prime }-{T_{3}}^{\prime }\right)-{F_{2}}^{\prime }=0,\\ \frac{\sqrt{3}}{2}\left(s_{0}\sin\delta_{p}+t_{0}\cos\delta_{p}\right)\left({T_{2}}^{\prime }-{T_{3}}^{\prime }\right)-\frac{3}{4}a\sin\delta_{p}\left({T_{2}}^{\prime }+{T_{3}}^{\prime }\right)=\frac{M}{b}. \end{array}$$

Combine equations (14) and (16); a quadratic equation about *s*_0_ similar to formula (21) can be received so as to find the value of *s*_0_ at this time.

### 4.3. Simulation Analyses

The parameters of the compression spring are shown in Table 1, where *l*_0_ is the original length of the spring, *h*_0_ is the spring pitch, *G* is the shear modulus, *E* is the elastic modulus, *r* is the spring radius, *d* is the diameter of the spring wire, and *K* is the spring elasticity coefficient. The moment of inertia *I* and bending stiffness of the spring can be calculated as *β*_0_, namely,

(25) $$\begin{array}{c} I=\frac{\pi d^{4}}{64}=3.068\times 10^{-11}{\text{m}}^{4},\\ \beta_{0}=\frac{2{EGIh}_{0}}{\pi r\left(E+2G\right)}=0.1609\text{N}\cdot {\text{m}}^{2}. \end{array}$$

The other parameters are *a* = 0.0965m, *b* = 0.084m, and *m* = 0.25kg. In practice, *t*_0_ is utilized to adjust the preload of three ropes; thereby, *t*_0_ is fixed at 0.062 m in simulation. By changing *δ*_*p*_ ∈ [0, *π*/9] and *δ*_*s*_ ∈ [0, 2*π*], the results are shown in Figure 11. Figures 11(a)–11(c) are the simulation curves of the rope length of three ropes, and Figures 11(d)–11(f) are the simulation curves of the tension of three ropes. As can be observed, when the length of the rope is small, the force exerted by the rope will be greater. Instead, when the length of the rope is large, the force exerted by the rope will be smaller; that is, the tension and length of each rope are complementary. Moreover, the length of the rope and the variation range of the tension are related to *δ*_*p*_. The larger the *δ*_*p*_ is, the larger the variation range of the rope length and tension is. This feature is consistent with the objective fact. When *δ*_*p*_ is constant, the curve of the length and tension of all ropes with the change of *δ*_*s*_ within 0 − 2*π* is symmetric. In order to get a better overview of this feature, as shown in Figure 12, the curves of the length and tension of the three ropes with the change of $\delta_{s}\in \left[\begin{array}{cc} 0, & 2\pi \end{array}\right]$ when *δ*_*p*_ = *π*/18 and *t*_0_ = 0.062mm are plotted.  Figure 12(a) shows the numerical curves curve of the length of three ropes, and Figure 12(b) shows the numerical curves of the tension of three ropes.

The article "Design and Analysis of a Flexible, Elastic, and Rope-Driven Parallel Mechanism for Wrist Rehabilitation" was published in 2020. Journal: Appl Bionics Biomech.

## 5. Workspace Analysis

The workspace is one of the important indexes to evaluate the performance of a robot. The analysis of the workspace is an important link in the design of the parallel mechanism. The workspace of the parallel mechanism designed in this paper is mainly related to the workspace of the flexible parallel mechanism. It refers to the set of center points of the moving platform with a group of positive rope tension that can make all the ropes in the tensioning state all the time by ignoring any external forces and torques on the mechanism. Furthermore, it is the area that the movable platform can reach under the condition of ensuring various rope tension. The characteristic is rope-driven. The rope can only bear the tension but not the pressure so that the binding force of the rope on the object can only be drawn along the straight direction of the rope, and its workspace is not in the joint limit range of the platform that can reach the point of the formation of the area. The actual workspace is much smaller than this area. Because the rope section is small, the binding force can be regarded as a concentrated force. Because of the unbearable pressure of the rope, the rope can only stop the movement trend of object elongation, but it cannot restrain the movement trend of object shortening. Therefore, the constraint that only restricts the unilateral motion of an object is called the unilateral constraint. The workspace of the wire-driven parallel mechanism must satisfy at least the following conditions [36, 37]. (a) The application of force and torque is not restricted. (b) The rope tension amplitude must be positive. (c) The rope force is between the preload and the maximum allowable tension. (d) Adequate stiffness of the structure should be ensured. (e) There is no singular configuration in the end effector. (f) The performance of rope interference does not happen.

The article "Design and Analysis of a Flexible, Elastic, and Rope-Driven Parallel Mechanism for Wrist Rehabilitation" was published in 2020. Journal: Appl Bionics Biomech.

The workspace of the flexible parallel mechanism is described by the motion range of the center point of the dynamic platform. The specific value and variation range are as follows: *δ*_*p*_ ∈ [0, *π*/9], *δ*_*s*_ ∈ [0, 2*π*], and *t*_0_ = 0.062. The software MATLAB is utilized to draw the workspace of the flexible parallel mechanism, as shown in Figure 13. It reveals that the workspace of the flexible parallel mechanism is in a parabolic shape, which is consistent with the objective facts.

## 6. Conclusions

This paper proposes a bionic flexible wrist parallel mechanism driven by rope and supported by compression spring to simulate the human wrist joint. The fixed base and moving platform of the parallel mechanism are connected by three ropes and a compression spring. A cylindrical compression spring is exploited to simulate the wrist support joints of human beings. The parallel mechanism is actuated and controlled by rope to simulate wrist muscles. The kinematic and static models of the system are built by the static equation and the lateral bending equation of the spring. The results of the simulation indicate that the kinematic and static models are reasonable and valuable. In order to obtain good motion performance, the workspace of the parallel mechanism is analyzed. The simulation results are reasonable, verifying that the design technique of the bionic flexible parallel joint mechanism and the novel method of workspace analysis are effective. The analytic method proposed in this paper will be helpful for analyzing the parallel mechanism with a flexible spine in the future. The results will play an important role in the reproduction of the human wrist movement and promote the development of a humanoid robot and rope-driven technology.

In future work, the optimization design of the rope layout will be paid attention to obtain the minimum rope driving force in the bionic flexible wrist parallel mechanism. This work will reduce the size of the driver and the cost. In this context, it is necessary to investigate the system dynamic model considering the flexible vibration and design the corresponding control strategy and space trajectory tracking control strategy of the bionic flexible wrist parallel mechanism.

## Figures and Tables

**Figure 1:** Freedom of movement of the wrist joint.

**Figure 2:** Structure of the flexible parallel mechanism of the wrist.

**Figure 3:** Structure of the adjustable handle part.

**Figure 4:** Structure of the flexible parallel mechanism.

**Figure 5:** Distribution and movement form of the cable restraint device.

The article "Design and Analysis of a Flexible, Elastic, and Rope-Driven Parallel Mechanism for Wrist Rehabilitation" was published in 2020. Journal: Appl Bionics Biomech.

**Figure 6:** Schematic diagram of the movement without the cable restraint device.

**Figure 7:** Schematic diagram of the movement with the cable restraint device.

**Figure 8:** Structure of the wrist fixing part.

**Figure 9:** Schematic diagram of the bionic flexible rope-driven parallel mechanism.

**Figure 10:** Force and torque balance system.

**Figure 11:** Inverse position and statics.

**Figure 12:** Curves of the rope length and tension when *δ*_*p*_ = *π*/18 and *t*_0_ = 0.062.

**Figure 13:** Workspace of the parallel mechanism.

**Table 1:** Parameters of compression coil spring.

*l*_0_ (m)	*h*_0_ (m)	*G* (GPa)	*E* (GPa)	*r* (m)	*d* (m)	*K* (N·m^−1^)
0.075	0.0124	73.94	193	0.063	0.005	4620

## Data Availability

The data is made available through the corresponding author's email or the first author's email.
